The article "Segmentation of Prefrontal Lobe Based on Improved Clustering Algorithm in Patients with Diabetes" was published in 2021. Journal: Comput Math Methods Med.

# Segmentation of Prefrontal Lobe Based on Improved Clustering Algorithm in Patients with Diabetes

**DOI:** 10.1155/2021/8129044

**Published:** 2021-10-07

**Authors:** Na Zhao, Qingzhen Zhao, Liang Wang, Xiuqing Wu, Rui Zhang, Haijun Feng

**Affiliations:** ^1^Department of Anesthesiology, The Affiliated Hospital of Medical School of Ningbo University, Ningbo 315020, China; ^2^Department of Anesthesiology, Affiliated Suzhou Science & Technology Town Hospital of Nanjing Medical University, Suzhou 215153, China

## Abstract

Diabetics are prone to postoperative cognitive dysfunction (POCD). The occurrence may be related to the damage of the prefrontal lobe. In this study, the prefrontal lobe was segmented based on an improved clustering algorithm in patients with diabetes, in order to evaluate the relationship between prefrontal lobe volume and COPD. In this study, a total of 48 diabetics who underwent selective noncardiac surgery were selected. Preoperative magnetic resonance imaging (MRI) images of the patients were segmented based on the improved clustering algorithm, and their prefrontal volume was measured. The correlation between the volume of the prefrontal lobe and *Z*-score or blood glucose was analyzed. Qualitative analysis shows that the gray matter, white matter, and cerebrospinal fluid based on the improved clustering algorithm were easy to distinguish. Quantitative evaluation results show that the proposed segmentation algorithm can obtain the optimal Jaccard coefficient and the least average segmentation time. There was a negative correlation between the volume of the prefrontal lobe and the *Z*-score. The cut-off value of prefrontal lobe volume for predicting POCD was <179.8, with the high specificity. There was a negative correlation between blood glucose and volume of the prefrontal lobe. From the results, we concluded that the segmentation of the prefrontal lobe based on an improved clustering algorithm before operation may predict the occurrence of POCD in diabetics.

## 1. Introduction

More and more evidence shows that the type 2 diabetes mellitus (T2DM) can cause damage to the function and integrity of brain tissue [1–4]. Cognitive damage is one of the manifestations of brain damage, and the damage of cognitive function is accompanied by the change of brain tissue structure [5, 6]. With the development of the course of disease, the cognitive impairment of T2DM can be manifested in various aspects, such as the decline of memory, attention, and learning ability, and gradually aggravate until dementia [7, 8].

Postoperative cognitive dysfunction (POCD) is a common complication of anesthesia operation [9], which often occurs in the elderly [10]. The incidence of POCD is higher because of the possible brain damage in diabetic patients [11]. POCD not only affects the patients' quality of life after operation but also leads to an increased incidence of postoperative pulmonary infection and death [12]. At present, there is no effective index to predict the occurrence of POCD [13].

The article "Segmentation of Prefrontal Lobe Based on Improved Clustering Algorithm in Patients with Diabetes" was published in 2021. Journal: Comput Math Methods Med.

The prefrontal cortex is located in front of the motor center of the body, which is the combined cortex of the frontal lobe. Research shows that the prefrontal lobe is closely related to cognitive function [14–17]. The results of neuroimaging show that the degree of prefrontal cortex atrophy can predict the change of cognitive function [18–20]. The improved clustering segmentation algorithm can effectively avoid the blindness of the initial cluster center selection and make the segmentation results faster and more accurate. Thus, the purpose of this study was to evaluate the accuracy of preoperative volume of the prefrontal lobe in magnetic resonance imaging (MRI) on predicting the occurrence of POCD in diabetics, in order to provide a reference for clinical practice.

## 2. Materials and Methods

### 2.1. General Information

In this study, 48 patients with T2DM who were 60-85 years old were enrolled in our hospital from January 2017 to December 2019. This study has been approved by the ethics committee of our hospital.

The inclusion criteria are as follows: (1) T2DM was diagnosed according to the diabetes diagnosis standard recommended by the WHO; (2) elective noncardiac surgery; (3) age from 60 to 85; (4) American Society of Anesthesiologists (ASA) levels I-III; and (5) informed consent by the patients.

The exclusion criteria are as follows: (1) preoperative depression or cognitive impairment; (2) drug abuse, alcohol abuse, or long-term use of benzodiazepines, antidepressants; (3) hearing or visual impairment; (4) cardiovascular and cerebrovascular accidents within 6 months or with neurological sequelae; (5) previous cardiac or central nervous system surgery; (6) emergency surgery or craniocerebral surgery; (7) illiteracy; and (8) have participated in other clinical studies.

### 2.2. Anesthesia Program

Before anesthesia, Atropine 0.5 mg and Phenobarbital 100 mg were intramuscularly injected. The invasive BP, HR, SpO_2_, and P_et_CO_2_ were monitored through catheterization of the radial artery, and the CVP was monitored catheterization of the right internal jugular vein. Auditory evoked potential index (AAI) was monitored by an A-line MLAFP ARX index monitor.

Anesthesia was induced by intravenous injection of midazolam 0.05-0.10 mg/kg, fentanyl 3-5 *μ*g/kg, vecuronium 0.1 mg/kg, and propofol 1.0-1.5 mg/kg. Mechanical ventilation was performed after tracheal intubation to maintain p-stare at P_et_CO_2_ 23-40 mmHg.

The article "Segmentation of Prefrontal Lobe Based on Improved Clustering Algorithm in Patients with Diabetes" was published in 2021. Journal: Comput Math Methods Med.

Anesthesia maintenance: inhalation of 1%~3% sevoflurane, intermittent intravenous infusion of fentanyl 2.5~5.0 *μ*g/kg·h, and intravenous vecuronium 0.025~0.050 mg/kg. When necessary, remifentanil 0.05~0.20 mg/kg·min and propofol 3~9 mg/kg·min were infused intravenously. When the MAP was less than 30% of basic value, intravenous ephedrine 5~10 mg/time was used. When the HR was less than 50 times/min, Atropine 0.2 mg/time was injected intravenously. The fluctuation of SP was kept within 30% of basic value, HR 50~100 times/min, AAI 15~25. After the operation, the patient will be sent back to the ward or intensive care unit according to the condition.

### 2.3. Cognitive Evaluation

Neuropsychological tests were conducted before and 4 days after the operation, including Wechsler adult memory, sensitive items in intelligence scale, connecting line, and nail board tests. The detailed test items were as follows:

1. Cumulative test: adding the same number (e.g., 3 or 4) to 49 continuously from 1, recording the time needed to complete and the number of errors and omissions, calculating rough scores according to the formula, this test content can reflect attention and calculation ability
2. Visual regeneration: allows the subjects to see 3 designed figures (a, b, and c) 10 s, and let them draw the figure and grade it according to the accuracy of the copied figure. This test content can reflect the ability of visual memory and the ability of visual-spatial analysis
3. Associative learning: designs a group of 10 pairs of words, reads them to the subjects in a specific order, writes them on 10 cards, and presents them to the subjects at the same time. The first word was read out by the tester, and the subject was asked to say another word according to his memory. The test was carried out three times in total, and the score was made according to the accuracy of the answer. This test content can reflect the language memory ability and visual memory ability
4. Digital breadth: this test includes two tests, consequent and reverse. Give the subject a group of numbers, and then, ask them to repeat the numbers with consequent and reverse direction. Score with the highest number of correct retelling. This test item can reflect the degree of concentration
5. Number sign: arranges a group of symbols and numbers, and then, the subjects match the numbers and symbols within 90 s and record the correct number. The correct number is the score. This test content can reflect the mental movement speed
6. Connecting line: allows the subjects to connect the numbers (including the numbers in upper and lower case) in order as soon as possible and record the required time. This test content can reflect the attention and mental movement speed
7. Nail board: insert a short stick on a special board by dominant hand and nondominant hand, respectively, and record the required time. This test content can reflect the fine movement speed

According to the occurrence of POCD, the patients were divided into the POCD group and the non-POCD group. The specific steps are as follows: (1) calculate the standard deviation(s) according to the first test result of the single test for the healthy elderly; (2) calculate the difference between the single preoperative test result and the postoperative test result of each patient (*X*_*i*_); (3) *Z*_*i*_ = *X*_*i*_/*s*, total *Z*‐score = *Z*_1_ + *Z*_2_ + +*Z*_9_; and (4) POCD occurs when total *Z*‐score ≥ 1.96.

The article "Segmentation of Prefrontal Lobe Based on Improved Clustering Algorithm in Patients with Diabetes" was published in 2021. Journal: Comput Math Methods Med.

### 2.4. Blood Glucose Test

All patients fasted after 8:00 p.m. for 3 consecutive days before operation; peripheral blood glucose was measured 7 times a day, i.e., before and after three meals and before sleep. Take the average blood glucose before three meals and bedtime as the average fasting blood glucose (FBI), and the average of blood glucose after three meals as the average 2 hours postprandial blood glucose (PBI).

### 2.5. Brain MR Image Segmentation Process

This paper presents an automatic segmentation algorithm for brain MR images. Firstly, color coding is applied to the source image to enhance the regions of interest in the image and make it easier to identify different tissues. Then, the initial clustering centers of white matter, gray matter, and cerebrospinal fluid regions are determined according to the anatomical prior knowledge and probability gray histogram; finally, the iterative operation is carried out according to the clustering segmentation algorithm, and the convergence is achieved when the set threshold is reached to complete the automatic image segmentation.

#### 2.5.1. Image Color Coding

Gray image is only represented by intensity values of 0-255, while color image can be represented by RGB color space. CIE LAB space is established on the basis of the international standard of color measurement formulated by the International Commission on lighting. It uses digital methods to describe human visual perception and can be converted into RGB color space. CIE LAB uses *b*, *a*, and *L* coordinate axes to define CIE color space, where image brightness *L*, the value range is [0,100], which means from pure black to pure white; chroma *a* means red-green axis, chroma *b* means blue-yellow axis, and the value range of them is [0, 10]. The image brightness is calculated by the YIQ color system formula and given by formula (1). The chromaticity value is obtained from the color spectrum of the source image.

(1) $$\begin{array}{c} L=B\times 0.114+G\times 0.587+R\times 0.299. \end{array}$$

The steps of image color coding are as follows: *I*, *I*_*C*_, and *I*_*T*_ are input gray image, source color spectrum image, and target image, respectively, and they have the same scale size; the corresponding image pixels are represented as *P*, *P*_*c*_, and *P*_*T*_.

1. The intensity *L* of gray image pixel *P* is obtained
2. The color spectral image pixel PC of the source image is obtained and converted into intensity *L*_*c*_ by formula (1)
3. The Euclidean distance formula is used to compare the intensities *L* and *L*_*c*_. Given by formula (2), gp and cp represent the number of pixels of the image, respectively

(2) $$\begin{array}{c} D=\left|L_{i}-L_{Cj}\right|,\;i=1,2,3\cdots gp,j=1,2,3\cdots cp \end{array}$$

(4) When 0 ≤ *D* ≤ 4, skip step (3); otherwise, convert *P* and *P*_*c*_ to CIE LAB color space

The article "Segmentation of Prefrontal Lobe Based on Improved Clustering Algorithm in Patients with Diabetes" was published in 2021. Journal: Comput Math Methods Med.

#### 2.5.2. Clustering Segmentation Algorithm

A clustering algorithm is an unsupervised model learning method [12], which can efficiently cluster large data and is widely used in image segmentation, pattern recognition, data mining, and other fields. The basic idea is as follows: select *K* objects as the initial clustering center; then, according to the clustering function, classify the sample points to the nearest cluster center, and update the new cluster center after adjustment; when the change range of two adjacent cluster centers is less than the set critical value, the clustering operation stops. The clustering objective function proposed in this paper is shown in formula (3). At this time, the image segmentation process is transformed into using the objective function to divide the voxels in the image into their categories.

(3) $$\begin{array}{c} R_{\left(z,k\right)}=\overset{m-1}{\underset{x=0}{\sum }}\overset{n-1}{\underset{y=0}{\sum }}\overset{k-1}{\underset{tc=0}{\sum }}\overset{z-1}{\underset{tp=0}{\sum }}\left|V_{\left(x,y,tp\right)}-C_{\left(z,tc\right)}\right|. \end{array}$$

When *z* > 1, 3D images can be processed, and when *z* = 1, they are applied to 2D images; **R**_(**z**, **k**)_ represents the number of initial clustering centers, that is, the number of segmented regions; **V**_(**x**, **y**, **tp**)_ represents the voxel value at the (**x**, **y**, **tp**) position in the image, **C**_(**z**, **tc**)_ represents the tc initial clustering centers on the *z* plane, and **V**_(**x**, **y**, **tp**)_ − **C**_(**z**, **tc**)_ represents the distance measure from the voxel **V**_(**x**, **y**, **tp**)_ to the clustering center **C**_(**z**, **tc**)_; *m*, *n* represents the size of each plane image.

The article "Segmentation of Prefrontal Lobe Based on Improved Clustering Algorithm in Patients with Diabetes" was published in 2021. Journal: Comput Math Methods Med.

#### 2.5.3. Initial Clustering Center Based on Gray Histogram

The selection of the initial cluster center has a great influence on the clustering results. If it is not selected properly, the global optimal classification results are hard to be obtained. In this paper, the image gray histogram is used to determine the initial clustering center. The gray histogram is given by

(4) $$\begin{array}{c} H_{z}=\overset{z-1}{\underset{p=0}{\sum }}\overset{n-1}{\underset{x=0}{\sum }}\overset{m-1}{\underset{y=0}{\sum }}g\left(z,x,y\right). \end{array}$$

The process of determining the initial cluster center can be explained by Figure 1. Firstly, the histogram of the source image is calculated, and then, the triangle is drawn to analyze the overlapping area, and the histogram curve is obtained. Finally, the initial clustering center point is obtained according to the intersection of the histogram curve. The specific steps are as follows:

1. Use formula (4) to traverse the histogram and detect all peak points

(5) $$\begin{array}{c} {HO}_{\left(z\right)}=\left\{H_{\left(z,i\right)}\;|\;H_{\left(z,i\right)}>H_{\left(z,i-1\right)},\;|\;H_{\left(z,i\right)}>H_{\left(z,i+1\right)},1《i《255\right\} \end{array}$$

(2) All peak points are screened by formula (6), and the peak points less than 5% of the maximum peak point are removed to get the peak point set PZ

(6) $$\begin{array}{c} P_{z}=\left\{\left(i\right)\;|\;\frac{{\text{HO}}_{\left(z,i\right)}}{{\text{HO}}_{\left(z,\max\right)}}>\frac{\left({\text{HO}}_{\left(z,\max\right)}\times 5\right)}{100},0《i《255\right\} \end{array}$$

(3) A new set of peak points is calculated by formula (7) to generate significant peak points in each region

(7) $$\begin{array}{c} {Pl}_{z}=\left\{P_{\left(z,i\right)}\;|\;P_{\left(z,i+1\right)}-P_{\left(z,i\right)}>10,0《i《255\right\} \end{array}$$

(4) Formula (8) is used to calculate the initial clustering center **C**_(**z**, **k**)_ of each region, in which **Range**_min(**z**, **k**)_ and **Range**_max(**z**, **k**)_ represent the smaller and larger range of each image plane *z*, respectively

(8) $$\begin{array}{c} C_{\left(z,k\right)}=\left\{{PI}_{\left(z,i\right)}\;|\;{Range}_{\min\left(z,k\right)}<{PI}_{\left(z,k\right)}《{Range}_{\max\left(z,k\right)}\right\} \end{array}$$

### 2.6. Evaluation of MRI

The 1.5T MRI machine (Siemens, Germany) was used to evaluate the volume of the prefrontal lobe. After the transverse, sagittal, and coronal stereoscopic localization was carried out, the frontal lobe area was scanned parallel to the line from anterior commissure to posterior commissure in the median sagittal plane (Figure 2).

The article "Segmentation of Prefrontal Lobe Based on Improved Clustering Algorithm in Patients with Diabetes" was published in 2021. Journal: Comput Math Methods Med.

In the transverse plane, adjust the appropriate window width and position, and use the mouse to draw the region of interest (ROI) of the prefrontal lobe boundary layer by layer. Because the frontal gyri were surrounded by cerebrospinal fluid, they can be semiautomatic identified by computer software. Thus, the key to delineate the frontal ROI was to determine the posterior boundary, which needs manual recognition. In order to unify the delineation of the posterior prefrontal boundary, the criteria for the demarcation of ROI in the frontal lobe were formulated with reference to the standard neuroanatomical atlas and under the guidance of neuroimaging and anatomists, the detail is shown in Figure 1.

In the three-dimensional (3D) reconstruction software, the prefrontal lobe and the whole brain's 3D image were reconstructed through the transverse plane, and the volume of the prefrontal lobe and brain is viewed and recorded through the property function (Figure 3). Then, the standardized volume of the prefrontal lobe = (measured volume of prefrontal lobe/volume of whole brain) × 1000.

### 2.7. Statistical Analysis

The SPSS 23.0 statistical software was used for the analysis of our biodata. The quantitative data were analyzed by the normality test. As the results were consistent with normal distribution, these data were expressed by $\bar{x}\pm s$. The data before and after operation were compared by the paired *t*-test, while the data in the POCD group and non-POCD were compared by Student's *t*-test. The qualitative data in various groups were compared by the chi-square test. The relationship between the volume of the prefrontal lobe and the *Z*-score or blood glucose was carried out by the Pearson correlation analysis. The receiver operator characteristic (ROC) curve was selected to calculate the cut-off value of prefrontal lobe volume, area under the curve (AUC), sensitivity, and specificity of volume of the prefrontal lobe for predicting POCD.

## 3. Results

### 3.1. Segmentation Results Based on Improved Clustering Algorithm

Qualitative analysis shows that the gray matter, white matter, and cerebrospinal fluid based on the improved clustering algorithm were easy to distinguish. Quantitative evaluation results show that the proposed segmentation algorithm can obtain the optimal Jaccard coefficient and the least average segmentation time (Table 1).

### 3.2. General Information and Intraoperative Index

In all the 48 diabetics, the POCD was found in 12 cases, and the incidence was 25%. The general information, including age, sex, body mass index (BMI), education level, and the intraoperative index, including ASA, operative time, anesthesia time, propofol dosage, sevoflurane dosage, and the use of vasoactive drugs, is shown in Table 2. There was no significant difference between the POCD and non-POCD groups (all *P* > 0.05), which indicated that the preoperative state of patients and the effect of anesthesia on the two groups were basically the same.

The article "Segmentation of Prefrontal Lobe Based on Improved Clustering Algorithm in Patients with Diabetes" was published in 2021. Journal: Comput Math Methods Med.

### 3.3. Neuropsychological Test

The detailed neuropsychological test results are shown in Table 3. The total *Z*-scores in the POCD and non-POCD groups were 3.0 ± 0.7 and 1.1 ± 0.5; the difference is statistically significant (*P* < 0.001). Compared with preoperative data, the postoperative cumulative test, visual regeneration, associative learning, and digital breadth (reverse) test were lower in the POCD group (all *P* < 0.05). In the non-POCD groups, only the cumulative test before and after operation has the statistical differences (*P* < 0.05).

### 3.4. Volume of the Frontal Lobe

The volume of the prefrontal lobe in the POCD group was 167.1 ± 16.6 cm^3^, while the volume of the prefrontal lobe in the non-POCD group was 196.0 ± 19.8 cm^3^. The volume of the prefrontal lobe in the POCD group was significantly smaller than the volume in the non-POCD group (*t* = 5.107, *P* < 0.001). There was a negative correlation between the volume of the prefrontal lobe and the *Z*-score (*r* = −0.324, *P* = 0.003). In the ROC curve, the cut-off value of the volume of the prefrontal lobe for predicting POCD was <179.8 (AUC = 0.859, *P* < 0.001), with the sensitivity, specificity, and Youden's index of 77.4%, 82.4%, and 0.598, respectively (Figure 4).

### 3.5. Blood Glucose

The FBI and PBI in POCD and non-POCD are shown in Figure 5. Compared with the non-POCD group, the FBI and PBI in the POCD group were relatively higher. There was a negative correlation between the volume of the prefrontal lobe and FBI (*r* = −0.418, *P* = 0.007) or PBI (*r* = 0.464, *P* = 0.012).

## 4. Discussion

In this study, there was no difference between the two groups in general and intraoperative conditions, which made the groups comparable. In this study, the AAI was maintained 15~25 during the operation, and the vital signs were stable. Thus, the effects of anesthesia depth and hemodynamic fluctuation on the test results were excluded [21].

The neuropsychological test used in this study shows that POCD has high specificity and sensitivity. The visual speech learning test and concept conversion task in the neuropsychological test methods (including 6 items) were recommended by the international organization for the study of postoperative cognitive impairment. The test and alphanumeric symbol test are basically similar to the associative learning test, online test, and digital symbol test [22]. The neuropsychological test used in this study can objectively reflect the cognitive function of the human brain.

The article "Segmentation of Prefrontal Lobe Based on Improved Clustering Algorithm in Patients with Diabetes" was published in 2021. Journal: Comput Math Methods Med.

In this study, parallel version is used to reduce the learning effect in the process of testing; each test is conducted by the same tester in the same environment and in the same time period to overcome the variability. It has been reported by foreign scholars that increasing the items of the neuropsychological test can not only improve the sensitivity of the test method but also significantly improve the false-positive rate [23]. The false-positive rate can affect the results of POCD-related studies, so that the results of similar studies are not comparable.

MRI has a good contrast resolution for soft tissue and multidirectional imaging characteristics [24]. It can clearly show the true anatomy section images of various layers of brain structure, because the volume of the prefrontal lobe can be affected by the volume of cranial content, which leads to the lack of comparability of data. In this study, the volume of the prefrontal lobe was standardized to eliminate the influence of the whole brain.

The results showed that the volume of the prefrontal lobe in the POCD group was smaller than that in the non-POCD group, and there was a negative correlation between the volume of the prefrontal lobe and the *Z*-score. The sensitivity, specificity, and Youden's index of predicting the occurrence of POCD were 77.4%, 82.4%, and 0.598, indicating that the preoperative volume of the prefrontal lobe measured in MRI can predict the occurrence of POCD. The cut-off value of frontal volume between patients with POCD and those without POCD was 179.8.

We further analyzed the relationship between blood glucose, volume of prefrontal, and POCD. The results showed that the FBI and PBI in POCD were significantly higher than the data in non-POCD, indicating that the high blood glucose is more likely to cause POCD. In addition, there was a negative correlation between the volume of the prefrontal lobe and FBI or PBI. Long-time hyperglycemia has damaged brain tissue, which is the morphological basis of POCD.

From our study, we implemented prefrontal image segmentation based on an improved clustering algorithm and used them in the prevention of POCD. However, we do not know the specific advantages of this method and other artificial intelligence algorithms [25, 26]. Reports also showed that different types of intracerebral hemorrhage can lead to changes in brain texture. So, whether POCD will cause brain texture changes is one of the directions we will consider in the future [27].

## 5. Conclusions

In conclusion, the segmentation of the prefrontal lobe based on an improved clustering algorithm before operation may predict the occurrence of POCD in diabetics. There was a negative correlation between blood glucose and volume of the prefrontal lobe. The reduction of the prefrontal lobe is related to the increase of blood glucose.

The article "Segmentation of Prefrontal Lobe Based on Improved Clustering Algorithm in Patients with Diabetes" was published in 2021. Journal: Comput Math Methods Med.

## Figures and Tables

**Figure 1:** Segmentation of the prefrontal lobe on the transverse plane. (a–c) Three typical transverse plane between the upper end of the frontal lobe to the lateral ventricle. Find the anterior central sulcus, along the deepest part of the sulcus, draw a straight line perpendicular to the longitudinal fissure of the brain. (d) Typical plane through the lateral ventricle. Draw along the anterior central sulcus to the front point of the lateral ventricle; then, draw a straight line to connect with the deepest point of the longitudinal fissure. (e) Typical plane through the lateral sulcus. Draw a line along the front of the lateral sulcus to the front point of the lateral ventricle. (f) Typical plane with the disappeared lateral ventricle. The lateral fissure was the posterior boundary of the prefrontal lobe and delineated along the boundary of the frontal lobe.

**Figure 2:** Localization of the prefrontal lobe: (a) transverse plane; (b) coronal plan; (c) sagittal plan; (d) median sagittal plane. The irregular shape area is the prefrontal lobe. The lines were the position of the typical transverse plane in the median sagittal plane.

**Figure 3:** Three-dimensional reconstruction of the prefrontal lobe and whole brain: (a) whole brain alone; (b) prefrontal lobe alone; (c, d) both the brain and the prefrontal lobe were shown.

**Figure 4:** The ROC curve of prefrontal lobe volume for predicting POCD.

**Figure 5:** The blood glucose in POCD and non-POCD groups.

**Table 1:** Average time-consuming results of different segmentation algorithms.

Item	Categories	Iterations	Jaccard coefficient	Average time
Multithreshold algorithm	4	1	0.347	1.709
Level set algorithm	0	1	0.546	2.894
*K*-means clustering	4	31	0.504	27.852
Improved clustering algorithm	4	1	0.886	0.142

**Table 2:** The general information and intraoperative index in two groups.

Item	POCD (*n* = 12)	Non-POCD (*n* = 36)	*t* or *χ*^2^	*P*
Age (year)	72.4 ± 6.8	71.6 ± 5.9	0.392	0.697
Sex (male/female)	8/4	19/17	0.705	0.401
BMI (kg/m^2^)	22.3 ± 2.1	21.4 ± 2.5	1.120	0.268
Education level (year)	6.7 ± 1.2	7.1 ± 1.4	0.886	0.380
ASA (II/III)	9/3	24/12	0.291	0.589
Operation time (min)	184.6 ± 45.2	192.5 ± 62.3	0.404	0.688
Anesthesia time (min)	214.3 ± 48.9	221.9 ± 51.2	0.450	0.655
Propofol dosage (mg)	289.4 ± 87.6	297.2 ± 92.8	0.256	0.799
Sevoflurane dosage (ml)	16.4 ± 5.2	17.3 ± 4.9	0.543	0.590
Vasoactive drugs (yes/no)	7/5	19/17	0.112	0.738

The article "Segmentation of Prefrontal Lobe Based on Improved Clustering Algorithm in Patients with Diabetes" was published in 2021. Journal: Comput Math Methods Med.

**Table 3:** The neuropsychological test in two groups (score).

Item	POCD (*n* = 12)	Non-POCD (*n* = 36)	*t*	*P*
Cumulative test				
Before operation	62.4 ± 21.2	73.1 ± 22.8	1.431	0.159
After operation	28.9 ± 13.7	61.4 ± 18.3	5.632	<0.001
*t*/*P*	4.598/<0.001	2.401/0.019		
Visual regeneration				
Before operation	10.4 ± 1.8	10.2 ± 2.1	0.295	0.769
After operation	8.1 ± 2.1	9.4 ± 1.8	2.079	0.043
*t*/*P*	2.881/0.009	1.735/0.087		
Associative learning				
Before operation	13.4 ± 2.3	13.6 ± 2.4	0.252	0.802
After operation	9.8 ± 2.6	12.5 ± 3.1	2.711	0.009
*t*/*P*	3.593/0.002	1.683/0.097		
Digital breadth (consequent)				
Before operation	5.7 ± 1.6	5.8 ± 1.4	0.207	0.837
After operation	5.5 ± 1.5	5.7 ± 1.1	0.497	0.622
*t*/*P*	0.316/0.755	0.337/0.737		
Digital breadth (reverse)				
Before operation	3.4 ± 0.9	3.3 ± 0.8	0.364	0.718
After operation	2.6 ± 0.8	3.1 ± 0.7	2.068	0.044
*t*/*P*	2.909/0.006	1.129/0.263		
Number sign				
Before operation	18.2 ± 3.7	17.4 ± 4.1	0.599	0.552
After operation	16.5 ± 2.8	16.2 ± 2.7	0.330	0.743
*t*/*P*	1.269/0.278	1.467/0.147		
Connecting line				
Before operation	62.8 ± 13.9	64.5 ± 15.4	0.339	0.736
After operation	64.2 ± 11.4	65.1 ± 16.8	0.172	0.864
*t*/*P*	0.270/0.790	0.158/0.875		
Nail board (dominant hand)				
Before operation	64.2 ± 11.8	62.3 ± 12.7	0.457	0.650
After operation	64.7 ± 12.1	62.1 ± 13.1	0.606	0.547
*t*/*P*	0.102/0.919	0.066/0.948		
Nail board (nondominant hand)				
Before operation	74.5 ± 15.9	73.2 ± 15.1	0.255	0.800
After operation	76.1 ± 11.6	75.8 ± 17.4	0.056	0.956
*t*/*P*	0.282/0.781	0.677/0.501		
Total *Z*	3.0 ± 0.7	1.1 ± 0.5	10.281	<0.001

## Data Availability

The data used to support the findings of this study are available from the corresponding author upon request.
